The article "Identification of novel candidate targets for suppressing ovarian cancer progression through IL-33/ST2 axis components using the system biology approach" was retracted in 2025. Reasons: duplicated images; overlap with earlier publications; concerns about the images; concerns about the authorship.

# Identification of novel candidate targets for suppressing ovarian cancer progression through IL-33/ST2 axis components using the system biology approach

**DOI:** 10.3389/fmolb.2023.1189527

**Published:** 2023-06-02

**Authors:** Geovanny Genaro Reivan Ortiz, Carmen Iulia Ciongradi, M. V. N. L. Chaitanya, Jayasankar Narayanan, Mohamed Mohany, Salim S. Al-Rejaie, José Luis Arias-Gonzáles, Ioan Sârbu, Marjan Assefi, Shaik Vaseem Akram, Yusuf Döğüş, Abolfazl Bahrami, Reza Akhavan-Sigari

**Affiliations:** ^1^ Laboratory of Basic Psychology, Behavioral Analysis and Programmatic Development (PAD-LAB), Catholic University of Cuenca, Cuenca, Ecuador; ^2^ Department of Surgery-Pediatric Surgery and Orthopedics, “Grigore T. Popa” University of Medicine and Pharmacy, Iași, Romania; ^3^ School of Pharmaceutical Sciences, Lovely Professional University, Phagwara, Punjab, India; ^4^ Department of Pharmacology, SRM Institute of Science and Technology, SRM College of Pharmacy, Kattankulathu, Tamil Nadu, India; ^5^ Department of Pharmacology and Toxicology, College of Pharmacy, King Saud University, Riyadh, Saudi Arabia; ^6^ Department of Social Sciences, Faculty of Social Studies, University of British Columbia, Vancouver, BC, Canada; ^7^ University of North Carolina, Greensboro, NC, United States; ^8^ Uttaranchal University, Dehradun, India; ^9^ Department of Medical Biochemistry, Faculty of Medicine, Cukurova University, Adana, Türkiye; ^10^ Biomedical Center for Systems Biology Science Munich, Ludwig-Maximilians-University, Munich, Germany; ^11^ Department of Neurosurgery, University Medical Center Tuebingen, Tuebingen, Germany; ^12^ Department of Healthcare Management and Clinical Research, Collegium Humanum Warsaw Management University, Warsaw, Poland

**Keywords:** IL-33, ST2, ovarian cancer, cancer-associated fibroblasts, MAPKs-NF-κB, gene expression, protein expression

## Abstract

**Background:** Cancer-associated fibroblasts (CAFs) of ovarian cancer (OvC) are the most prevalent element of the tumor microenvironment (TM). By promoting angiogenesis, immunological suppression, and invasion, CAFs speed up the growth of tumors by changing the extracellular matrix’s structure and composition and/or initiating the epithelial cells (EPT). IL-33/ST2 signaling has drawn a lot of attention since it acts as a pro-tumor alarmin and encourages spread by altering TM.

**Methods:** Differentially expressed genes (DEGs) of the OvC tumor microenvironment were found in the GEO database, qRT-PCR, western blotting, and immunohistochemistry, and their presence and changes in healthy and tumor tissue content were examined. Primary cultures of healthy fibroblasts and CAFs obtained from healthy and tumor tissues retrieved from OvC samples were used for *in vitro* and *in vivo* investigations. Cultured primary human CAFs were utilized to investigate the regulation and the IL-33/ST2 axis role in the inflammation reactions.

**Results:** Although ST2 and IL-33 expression was detected in both epithelial (EPT) and fibroblast cells of ovarian cancer, they are more abundant in CAFs. Lipopolysaccharides, serum amyloid A1, and IL-1β, the inflammatory mediators, could all induce IL-33 expression through NF-κB activation in human CAFs. In turn, via the ST2 receptor, IL-33 affected the production of IL-6, IL-1β, and PTGS2 in human CAFs via the MAPKs-NF-κB pathway.

**Conclusion:** Our findings suggest that IL-33/ST2 is affected by the interaction of CAFs and epithelial cells inside the tumor microenvironment. Activation of this axis leads to increased expression of inflammatory factors in tumor CAFs and EPT cells. Therefore, targeting the IL-33/ST2 axis could have potential value in the prevention of OvC progression.

## 1 Introduction

Ovarian cancer (OvC) is the most malignant reproductive tumor in women worldwide (Li et al., 2018). In 2018, there were 14,070 fatalities and an estimated 22,240 new cases in the United States (Siegel et al., 2018). The majority of OvC patients currently undergo chemotherapy using platinum/paclitaxel-based regimens after tumor reduction surgery; nonetheless, chemoresistance frequently arises, leading to failure of treatment and a casualty rate of more than 90% (Agarwal and Kaye, 2003). In order to clinically control ovarian cancer, medical oncologists may benefit from a better knowledge of the disease pathophysiology and the identification of new therapeutic targets. Some cells, including recruited macrophages/lymphocytes, epithelial cells, cancer-associated fibroblasts, endothelial cells, and tumor cells, make up the complex structure known as the tumor microenvironment. These cells communicate with one another and with the tumor cells through the use of cell–cell communication and soluble elements (Whiteside, 2008; Pietras and Ostman, 2010). An immune response can delay or accelerate the progression of a tumor relying on the situation and predominant profile of cytokine (Swartz et al., 2012; Landskron et al., 2014). A fibrotic response of some tumors was also noted. Cancer-associated fibroblasts (CAFs) are the considerable prevalent stromal cells among all cell types which drive a fibrotic response to a long-term environment of the inflammation (Rybinski et al., 2014). With the release of cytokines, soluble components of the tumor microenvironment (TM) can also stimulate cell invasion. The IL-33/ST2 pathway has recently attracted a lot of attention as an alarmin of pro-tumor that accelerates metastasis by causing alterations in the TM.

Interleukin-33 (IL-33) is an interleukin superfamily member that can operate both as a chromatin-associated factor and as an alarmin cytokine regulating gene transcription (Bertheloot and Latz, 2017; Cayrol and Girard, 2018; Cayrol and Girard, 2022). As an alarmin cytokine, upon cell damage or injury, IL-33 is secreted into the extracellular environment and interacts with its distinctive receptor ST2 (suppression of tumorigenicity 2), which exists in two differentially spliced forms, namely, the membrane-bound genuine ST2 receptor that mediates IL-33 cytokine activities and a soluble receptor (sST2) that inhibits IL-33 bioactivities (Griesenauer and Paczesny, 2017). The membrane-bound ST2 is associated with the IL1R/toll-like receptor family (Chackerian et al., 2007), which can activate intracellular signaling consisting of MAPK (mitogen-activated protein kinase) and NF-κB (nuclear factor-kappa B) pathways to participate in both chronic and acute inflammatory disorders (Miller et al., 2017; Huang S et al., 2018; Vasanthakumar and Kallies, 2019; Huang et al., 2021; Miller et al., 2022). It is discovered that ST2 and IL-33 are produced in different cell types, including immunocytes, mesenchymal cells, endothelial cells, and epithelial cells (Moussion et al., 2008; Hu et al., 2014; Saied et al., 2017; Chen et al., 2018). Current research has indicated that ovarian cancer tissues and tumor metastatic lesions exhibit significantly higher levels of ST2 receptor and IL-33 gene expression than normal ovarian tissues. Moreover, compared to benign ovarian tumors, mucinous and serous ovarian cancers express IL-33 at a considerably higher level, which raises the tumor grade. According to other studies, epithelial ovarian cancer patients’ shorter survival times are correlated with higher IL-33 and ST2 expression (De la Fuente et al., 2015; Tong et al., 2016). Both the ST2L (membrane-anchored) and sST2 (soluble form) receptors with anti-inflammatory capabilities are produced by IL-33 (Chen et al., 2013). Furthermore, in some cancer patients, CAFs’ produced IL-33 which has been linked to invasion via promoting the epithelial–mesenchymal transition (EMT) (Lili et al., 2013), underscoring the significance of researching IL-33 in metastasis. However, it is unknown whether CAFs, the reservoir of multiple inflammatory signaling molecules, can also express IL-33 and ST2 to participate in OvC.

In this study, by focusing directly on OvC datasets, we also addressed this issue by exploring cell-specific expression patterns of ST2 and IL-33 genes and proteins in CAFs of ovarian cancer. Furthermore, we investigated the effect of some products including lipopolysaccharide (LPS), acute-phase protein serum amyloid A1 (SAA1), and JSH-23 as an inhibitor of NF-κB, IL-1β, and IL-33 itself on IL-33 expression in ovarian CAFs. Moreover, the role of ST2 and IL-33 in the regulation of pivotal inflammatory molecules pertinent to OvC, such as COX-2 (cyclooxygenase-2), p38, IL-1β, p65, and IL-6, the rate-limiting enzyme applied in the underlying intracellular signaling pathways, was also investigated in ovarian cancer progression and histopathological/clinical features.

## 2 Materials and methods

### 2.1 Data sources and genes expression analysis

We retrieved mRNA-expression data sets from the GEO (Gene Expression Omnibus) database. Inclusion data of this study for bulk or single-cell dataset selection were as follows: OvC-related mRNA data included GSE38666 (Huang C et al., 2018), GSE73064 (Gao et al., 2019), GSE126378 (Goossens et al., 2019), GSE138072 (Fan et al., 2020), GSE155164 (Odunsi et al., 2022), GSE147082 (Olalekan et al., 2021), GSE203612 (Barkley et al., 2022), GSE211687 (Garsed et al., 2022), and GSE180661 (Vázquez-García et al., 2022). In this work, we used 814 samples of patients and healthy tissues. Utilizing the ComBat-seq package (R package), the batch effects of the different RNA-seq data were eliminated (Leek et al., 2012). The original sequence was filtered and washed utilizing Seqtk software, and the “N”-containing, low-quality reads, and linker sequence were filtered out of the raw data obtained by sequencing. The data quality was assessed utilizing FastQC. Using HISAT 2.0, the filtered clean reads were mapped to the *Human sapiens* reference genome (Kim et al., 2015). By calculating the FPKM value with the help of edgeR, each gene expression level was normalized. The outcomes were differently screened, and FDR and fold change parameters were utilized to estimate them. In this work, the thresholds for substantial differential expression were FDR <0.05 and logFC (|log2 (FC)| > 1.5).

### 2.2 Gene Ontology and KEGG analysis

The GOseq R program was utilized to implement the GO enrichment analysis of differentially expressed genes (DEGs) (Chin et al., 2014). GO terms were enriched in the recognized biological processes utilizing GO enrichment analysis. To achieve significantly enriched Gene Ontology terms for DEGs, all DEGs were mapped to the Gene Ontology database (http://www.geneontology.org/), and the gene numbers were computed for each term using the hypergeometric assay. These terms have then resembled the genomic background. GO keywords were deemed to be significantly enriched by DEGs if their corrected *p*-values were less than 0.01. The pathway enrichment analysis and statistical testing of the differentially expressed mRNAs in KEGG (http://www.genome.jp/kegg/) were carried out using KOBAS software.

### 2.3 PPI evaluation

Tools for comprehending protein interactions include GeneMANIA and the STRING database (http://string-143db.org/and https://genemania.org/, respectively). We entered the differential genes into the STRING database and computed the protein–protein interaction relationship. The screening condition was established at a confidence level of >0.4 and a degree of >1. Finally, Cytoscape software was used to detect modules and hubs using the calculation results from the databases (Bader and Hogue, 2003; Sherman et al., 2007; Bindea et al., 2009).

### 2.4 Estimation of the TM cell infiltration

The immune score, stromal score, ESTIMATE score, and tumor purity for tumor samples were estimated using the R package ESTIMATE (Newman et al., 2015). Meanwhile, the levels of infiltrating cancer-associated fibroblast and epithelial cells were calculated by EPIC, MCP counter, and tumor immune dysfunction and exclusion (TIDE), and those of other immune cells were calculated by CIBERSORT, EPIC, TIMER, and MCP counter algorithms in the TM of ovarian cancer (Becht et al., 2016; Li W et al., 2017; Racle et al., 2017; Jiang et al., 2018).

### 2.5 Patients

All experimental protocols were approved by the Institutional Review Boards (IRBs) of the two study sites. The institutional review board of King Abdulaziz Medical City (IRB approved: protocol number study: IRB- BC-881-23) and King Fahad Specialist Hospital (IRB approved: protocol number study: IRB-OCD0348) approved this study by following the ethical standards and the Helsinki Declaration. Informed consent(s) was obtained from patients or their legal guardian(s). Tissue samples between 2015 and 2021 were collected in designated collection media at the time of surgery under the guidelines of the pathology departments following relevant guidelines and regulations. We included 172 samples from consecutive consented patients (average age 54.3 ± 12 years old) with ovarian tumors at any stage/grade of the disease undergoing surgery with or without pre-treatment/history of any previous carcinoma. Both tumor and healthy tissue were obtained as provided by the two pathologists, depending upon the availability of the tissue on a case-to-case basis. Therefore, the pathologists from each center worked together to macroscopically choose tumor samples, including the invasive front and core, and normal ovarian tissues, immediately following surgery. This was carried out to ensure homogeneity between samples. Each chosen tissue provided a little fragment, which was then kept at −80°C until it was later delivered to the laboratory for further analyses. For immunohistochemical examination, healthy and tumor biopsy samples were embedded in paraffin and fixed in 24% paraformaldehyde. For immunofluorescence investigation, healthy and tumor histology sections were also used. Following the signing of an informed permission form, samples of plasma from 56 age-matched healthy and OvC patients were collected. For association analysis, clinical information from OvC patients and controls was also gathered. The demographic features of recruited women are shown in Supplementary Table S1.

### 2.6 Isolation of cancer-associated fibroblast and epithelial cells

All primary cells obtained from surgical tissues were subjected to CAFs isolation using anti-fibroblast magnetic microbeads (Miltenyi Biotech, Cologne, Germany). Briefly, 1 × 10^6^ cells were centrifuged at ×300g for 10 min. Cell pellets were then resuspended in 100 μL of buffer containing a final concentration of 0.5% bovine serum albumin and 2 mM ethylenediaminetetraacetic acid dissolved in pH 7.2, calcium- and magnesium-free phosphate-buffered saline and incubated with 20 μL of human anti-fibroblast microbeads antibody (Miltenyi Biotec, CA, United States) for 1 h. Cells were then separated using a MiniMACS™ cell separator (Miltenyi Biotec, CA, United States). Isolated cells were then continued to be cultured in the media consisting of RPMI1640 (Life Technologies, NY, United States) supplemented with 10% fetal bovine serum (FBS) (Life Technologies, NY, United States) and 1% penicillin/streptomycin (Life Technologies, NY, United States). The epithelial cell population was also obtained by the similar method, using the human EpCAM magnetic microbeads antibody (Miltenyi Biotec, CA, United States). The purity of epithelial cells and CAFs was monitored by testing the expression of markers by qRT-PCR and immunocytochemistry. Briefly, RNA extraction was performed using the Qiagen RNEasy MiniKit and Qiashredder Kit according to the manufacturer’s (Qiagen, Germantown, MD, United States) protocol. Cells were released from the culture and pelleted by centrifugation at 1,500 rpm for 5 min. Cells were placed in lysis buffer and lysed using the Qiashredder system. RNA was then extracted using appropriate reagents. qRT-PCR was performed using the Roche LightCycler96 platform. In brief, appropriate primers for each marker of interest were mixed with Roche FastStart Essential DNA Green Master Mix and added to a 96-well plate. Each sample was run in triplicates (Roche LightCycler 96 Software version 1.1). Appropriate primers for each marker were ordered from Integrated DNA Technologies. The list of primers related to negative and positive expression of CAF and EPT markers is shown in Supplementary Table S2. Immunofluorescence staining for CAF and EPT of samples were fixed with 4% paraformaldehyde and incubated with α-SMA (rabbit monoclonal; 1:100; Abcam, Cambridge, United Kingdom), FSP-1 (rabbit monoclonal; 1:100; Abcam, Cambridge, United Kingdom), FAP (rabbit monoclonal; 1:100; Abcam, Cambridge, United Kingdom), CK8 (rabbit monoclonal; 1:100; Abcam, Cambridge, United Kingdom), E-cadherin (rabbit monoclonal; 1:100; Abcam, Cambridge, United Kingdom), and EpCAM (rabbit monoclonal; 1:100; Abcam, Cambridge, United Kingdom) overnight at 4°C. CAFs were then incubated with associated Alex Fluor 594-conjugated anti-rabbit IgG for 1 h. Nuclei were counterstained with DAPI.

### 2.7 ELISA assay

Levels of IL-33 and sST2 were measured by the enzyme-linked immunosorbent assays (ELISA) in the CAFs and EPT. For sST2 estimation, we used the Human ST2 ELISA Kit (Biorbyt Ltd., Cambridge, United Kingdom, product number: orb219434), and for the measurement of IL-33, the Human IL-33 ELISA Kit (Biorbyt Ltd., Cambridge, United Kingdom, product number: orb390944) was used. The related cells were formalized on ice in order to accumulate for centrifugation at 3,000 g for 25 min to detect IL-33 and sST2, in the supernatant. Utilizing an ELISA reader and ELISA assay (ShengGong Biological Technology, Shanghai, China), the levels of IL-33 and sST2 were detected. Each experiment was carried out three times.

### 2.8 RNA extraction

Utilizing an RNA extraction kit (OMEGA Bio-Tek), whole RNA was extracted from ovarian tissue taken from the tumor and healthy surrounding tissues. Utilizing an Agilent 2,200 TapeStation and a NanoDrop, RNA integrity and purity were assessed after extraction using the following parameters: an RNA integrity number value of 7.0, a ratio of A260/A230 equal 2.0, and a ratio of A260/A280 equal 1.8.

### 2.9 Measurement of IL-33 and ST2 abundance in CAFs with qRT-PCR and WB

Utilizing a Prime-Script RT Kit, reverse transcription was performed after RNA concentration, and quality was assessed (TaKaRa, Kyoto, Japan). qRT-PCR was utilized to quantify *IL-33*, *ST2,* and inflammatory genes expressions following the aforementioned power SYBR^®^ Premix TaqTM and reverse-transcribed cDNA. For the loading control, β-actin (housekeeping gene) was amplified simultaneously. The 2^−△△Ct^ calculation was utilized to quantify the relative expression of the gene. Supplementary Table S3 provides the qRT-PCR primer sequences. Total cellular protein was extracted from the frozen ovary samples with a radioimmunoprecipitation assay lysis buffer (RIPA) including inhibitors for phosphatase and protease (Roche, Indianapolis, IN). Using the Bradford method for measuring the protein concentration, WB was used to ascertain IL-33 and ST2 protein levels. A polyacrylamide gel was used to electrophorese 25 μg of protein. After being transferred to a nitrocellulose membrane blot, it was then intercepted with 4% non-fat milk and incubated with antibodies against ST2 (1:500; PTMab) and IL-33 (1:1000; GeneTex) for an overnight period at 4°C. Next, it was incubated with the related secondary antibodies conjugated with peroxidase of horseradish. A G-Box chemiluminescence picture-taken device was exploited to develop the peroxidase activity utilizing a chemiluminescence detection technique. By scanning the same blot with an anti-actin antibody (1:1000; Proteintech), an internal loading check was carried out. Protein abundance was determined by comparing the band intensity of ST2 or IL-33 to that of β-actin.

### 2.10 Genetic alteration and ChIP assay

We used the cBioportal tool (http://www.cbioportal.org/) to calculate the IL-33 alteration frequency and gene mutation profile in cancer patients (Gao et al., 2013). Microsatellite instability (MSI) is associated with nucleotide insertions and deletions in the microsatellite loci (Knijnenburg et al., 2018). Formaldehyde (Sigma-Aldrich) was used to cross-link the spinal cord cells of mice for 10 min at a temperature of 37°C. Using a commercial kit (Beyotime, China), the chromatin immunoprecipitation (ChIP) test was conducted based on the instructions of the manufacturer. Santa Cruz Biotechnology provided control normal IgG and the acetyl-histone H3/H4 antibodies. Using primers designed specifically for the PCR Master Mix and the promoter of the IL-33 and ST2 genes (Beyotime, China), ChIP-purified DNA was performed using a conventional polymerase chain reaction. PCR outcomes were isolated into 2 %agarose gels following the PCR reaction, and Tanon’s gel imaging system software was used to detect the results. Utilizing the cycle threshold (Ct), specific enrichment is calculated as follows: 2(Ct of control ChIP-Ct input)/2(Ct of AcH3/H4 ChIP-Ct input).

### 2.11 IL-33 and ST2 immunohistochemical staining

The ovary tissue from the tumor and healthy surrounding tissues were fixed at 12% paraformaldehyde and entrenched in paraffin for sectioning for immunohistochemical dying. This allowed researchers to observe the distribution of ST2 and IL-33 in human ovary tissue. Incubation with the primary antibody against IL-33 (1:500; GeneTex) or ST2 (1:500; R&D systems) or related non-immune serum (Proteintech) as control was performed on the section behind deparaffinization and slaking the peroxidase action with 0.4% H_2_O_2_. After washing, the partition was treated with the avidin-biotin complex and a biotinylated antibody coupled with peroxidase of horseradish. The agent 3-amino-9-ethyl carbazole was used to create the peroxidase action, which produced red color. The slide was inspected using a standard bright field microscope after being counterstained with the blue color hematoxylin (Zeiss).

### 2.12 Indirect immunofluorescence

The co-expression of ST2/E-cadherin and IL-33/α-SMA in paraffin histological partitions from the healthy and tumor samples was evaluated using immunofluorescence. In a nutshell, Merck KGaA NeoClear was used to deparaffinize the sections, and then a variety of alcohols, ranging from 99% to 65% ethanol, was used to rehydrate them. The antigenic healing was performed using sodium citrate with pH = 6 for ST2/Ecad and EDTA with pH = 7.5 for IL-33/-SMA. In 2x PBS containing 2% normal donkey serum, 4% bovine serum albumin (BSA), and 150 mM glycine, the sections were then treated (for non-specific protein plugging and autofluorescence, respectively). The compartments were incubated for an hour at 37˚C with the primary antibodies including anti-α-SMA (1/500), anti-IL-33 (1/500), anti-ST2 (1/1,000), monoclonal mouse antibody (Sigma-Aldrich), and polyclonal goat antibody (R and D Systems). After tissue slices had been rinsed in PBS for an hour at 37˚ C, secondary antibodies were added. Hoechst 33,342 (1/1,000) was operated to create nuclear counterstain. Lastly, a coverslip and mounting solution were used to cover the slides (Dako). The confocal microscope was utilized to view the slides at ×60 and ×20 magnifications.

### 2.13 Treatment of cancer-associated fibroblasts

To evaluate the ST2 and IL-33 expression between epithelial cells and CAFs, the cells were cultivated for 4 days and then prepared for gene and protein extractions and expression analyses. To study the regulation of IL-33 expression and the IL-33 effect on inflammatory molecules, CAFs were cultivated for 4 days before reagent antidote were used in FBS- and phenol-red-free DMEM. To examine the regulation of IL-33 expression in fibroblasts, the cells were treated with LPS (0, 1, 10, and 50 ng/mL; Sigma; 24 h), IL-1β (0, 0.1, 1, and 10 ng/mL; Sigma; 24 h), SAA1 (0, 1, 10, and 50 ng/mL; PeproTech; 24 h), and IL-33 (50, 100, and 200 ng/mL; 8 h). To investigate the NF-κB role in the IL-33 regulation, the cells were treated with SAA1 (50 ng/mL; 24 h), LPS (10 ng/mL; 24 h), IL-33 (100 ng/mL; 8 h), and IL-1β (10 ng/mL; 24 h), in the absence or presence of JSH-23 (10 μM; Selleck, Houston, TX), an inhibitor of NF-κB. To examine the IL-33 effect on the COX-2, IL-6, and IL-1β expression, concentration-dependent and time course analyses were performed. For time course analysis, CAFs were treated with IL-33 (100 ng/mL) for 2, 4, 8, 12, and 24 h. For the concentration-dependent analysis, CAFs were treated with IL-33 for 8 h at 50, 100, and 200 ng/mL concentrations. To study the IL-33 (100 ng/mL) effects on the phosphorylation of MAPKs (JNK, p38, and ERK1/2) and p65, a subunit of NF-κB, a time course study (0.5, 1, 2, 4 and 6 h) was performed. To explore the involvement of the MAPKs pathway in the p65 phosphorylation and the regulation of IL-6, COX-2, and IL-1β by IL-33, CAFs were treated with IL-33 (150 ng/mL) for 8 h in the lack or existence of the JNK inhibitor SP600125 (10 μM), the ERK1/2 inhibitor PD98059 (20 μM), and the p38 inhibitor SB203580 (10 μM). To study the NF-κB involvement in the COX-2, IL-6, and IL-1β induction by IL-33, CAFs were treated with IL-33 for 8 h in the lack or existence of JSH-23 (10 μM). To explore the ST2 involvement in the inactivation of MAPKs and NF-κB, and in the IL-6, IL-1β, and COX-2 induction by IL-33, CAFs were treated with IL-33 in the lack or existence of small interfering RNA (siRNA) moderated ST2 knockdown. All inhibitors were added 1 h before IL-1β, LPS, and SAA1 for IL-33 treatment. After that, the conditioned cultural medium was managed for the secreted IL-6, IL-1β, and PTGS2 measurement with enzyme immunoassay (ELISA) kits (Proteintech) following the manufacturer’s instruction. IL-33 in the conditioned medium was measured with western blotting after concentrating with a centrifugal filter device (Millipore) following manufacturer’s instructions as expressed earlier (Wang et al., 2019). The cells were prepared for the whole protein and RNA extraction for investigations of COX-2, IL-6, IL-1β, and IL-33 protein and gene expressions with western blotting and qRT-PCR, respectively.

### 2.14 siRNA transfection in CAFs with electroporation

To investigate the ST2 role in mediating the effects of IL-33, siRNA-mediated knockdown of ST2 was performed. After separation, CAFs were electroporated utilizing an electroporator at 170 V for 5 m with 50 nM of siRNA (5′-GCA​GCC​AAG​AAC​TGA​GTG​CCT​T-3′) against ST2. Prior to receiving the IL-33 therapy, the cells were cultivated for 72 h in DMEM having 12% FBS. Western blotting and qRT-PCR were utilized to evaluate the knockdown efficacy.

### 2.15 Gene and protein expression analyses from CAFs

Utilizing qRT-PCR, the mRNA abundance of PTGS2, COX-2, ST2, IL-6, and IL-33 was assessed. As a loading control, the common GAPDH gene was amplified concurrently. The RIPA lysis buffer with inhibitors of protease and phosphatase was used to recover cellular protein. According to the procedure outlined previously, the protein expressions of ST2, IL-33, p38, COX-2, p-p38, p-p65, p65, p-JNK, JNK, p-ERK, and ERK were evaluated using western blotting. Loading controls were conducted by exploring the blot with an antibody of GAPDH for the concentrated conditioned culture medium. The direct antibodies utilized for WB in this analysis were included ST2 (1; 1,000; PTMab), phosphorylated p38 (1:500; GeneTex), p38 (1:500; PTMab), phosphorylated ERK1/2 (1:500; GeneTex), ERK1/2 (1:500; GeneTex), JNK (1:1,000; GeneTex), phosphorylated JNK (1:1,000; GeneTex), p65 (1:1,000; GeneTex), phosphorylated p65 (1:1,000; GeneTex), PTGS2 (1:1,000; GeneTex) (all from Cell Signaling, Danvers, MA), IL-33 (1:1,000; GeneTex), and GAPDH antibody (1:10,000; Proteintech).

### 2.16 Cell culture and cell lines

King Abdulaziz Hospital got the human ovarian cancer, Caov-3, and SK-OV-3 cell lines from the Chinese Academy of Sciences. Both lines were kept alive under conventional cultural requirements (37°C, 4% CO_2_) in DMEM containing 12% FBS.

### 2.17 Cell viability assay

Cell counting kit-8 (CCK-8) tests were used to measure cell proliferation, as previously reported (Wang et al. 2018). In 96-well plates, cells at a dilution of 5 × 10^3^ were incubated for 0, 24, 48, or 72 h before CCK-8 was used following the manufacturer’s instructions. Cell viability was assessed using the triplicate optical density reading after 4 h of CCK-8 incubation.

### 2.18 Wound healing assay

Wound healing experiments were conducted to measure cell migration (Eoh et al., 2018). On 6-well plates, cells (5 × 10^4^ per well) were kept alive. Cells were harvested at 90% confluence using a 200-L pipette tip to make a small incision area. Following two rounds of phosphate-buffered saline washing, the cells underwent a 24-hour incubation period in DMEM at 4% CO_2_ and 37°C. Images were taken at the appropriate intervals, and ImageJ was used to calculate the wound’s width. The average of separate test data was calculated and represented as an original width percentage after 10 measurements were taken along the length of the incision at random intervals.

### 2.19 Invasion assay

At 5 × 10^4^ cells per well density, cells were separated into the top Transwell section with 6-meter pores. In 24-well plates containing 20% FBS, sections with the Matrigel matrix for testing migration or invasion of cells were raised. Without the use of FBS, cells were grown inside the section. Following 24 h, cells that had invaded or migrated and were sticking to the lower section area were fixed and dyed with 6% crystal violet. In 12 microscope domains for each well, cells were counted.

### 2.20 Statistical analysis

The means and SEM for all data are presented. Repeated tests using various ovary tissues obtained from independent patients are indicated by the number for each experiment. When necessary, one-way ANOVA, Student's t-tests, and Mann–Whitney U were carried out after the use of the Shapiro–Wilk normalization test. These tests were then pursued by the Newman–Keuls multiple comparison test. The thresholds for statistical significance were *p* < 0.01 and *p* < 0.05.

## 3 Results

### 3.1 Analysis of differentially expressed genes

In total, 12,216 and 16,117 mRNAs were detected in the healthy and patient groups, respectively. The maximum values of FPKM in the two groups were 0.89 × 10^4^ and 1.31 × 10^4^, and the minimum values were 2.98 × 10^−3^ and 3.22 × 10^−3^, respectively. The aforementioned results indicate that the healthy group expressed fewer genes than the patient group, and the magnitude of gene expression was also lower (average and peak) in the healthy group. 1,602 mRNAs were detected according to |log2FoldChange|>1.5 and *p* < 0.05 when transcriptome data of the two groups were compared. From these, 1,141 (71.22%) and 461 (28.78%) DEGs were upregulated and downregulated, respectively (Supplementary Table S4). All DEGs (volcano plot) are shown in Figure 1A. Using comprehensive clustering of MCODE, a core module with 49 genes was clustered (Supplementary Table S5).

**FIGURE 1:** Identification of differential expression genes (DEGs). **(A)** Volcano plot of DEGs between patient and healthy groups. **(B)** Heatmap showing detailed pathways and OvC samples. **(C)** GSEA plot detecting the relevant pathways between OvC and healthy samples.

### 3.2 Biological pathways enrichment analysis

Using pathway analysis, the DEGs were enriched in a total of 46 signaling pathways, including the FOXO pathway, MAPK pathway, cytokine-cytokine receptor, JAK-STAT pathway, the NF-κB pathway, TNF pathway, endometrial cancer pathway, fructose and mannose metabolism, IL-17 pathway, toll-like receptor pathway, NOD-like receptor pathway, and cAMP pathway (Figure 1B). Next, the top 14 hub genes were filtered which included IL-33, IL-17, FOXO1, IL-6, COX-2, MAPK3, CDK4, CDK2, MAPK14, AKT1, ERK1, PLK1, TNF-α, and TLR2 genes. In addition, the significantly enriched pathways for OvC included apoptosis, inflammatory response, MAPK signaling, FOXO signaling, TNF-α signaling, and IL-33 signaling via NF-κB, which is shown through the GSEA plot (Figure 1C).

### 3.3 Investigating the relevance between CAF signatures and components as well as signals in OvC immune microenvironment

Given the impressive ability of CAF signatures to distinguish between patients with widely varying outcomes, the role of CAFs in the prognosis of OvC patients deserves further exploration. The relevance of CAFs to prognosis should be demonstrated with more proof. Prognostic-oriented clustering in the OvC integrated cohort exhibited distinct CAF signatures and hub genes between the groups (Figure 2A). As a prominent population in the TM of OvC, CAFs undeniably engage in shaping the immune microenvironment. Thus, we demonstrated correlations between CAF signatures with cytokines including interleukins and chemokines, in which IL-33 and CCL11 were remarkable because of their apparent positive correlations with CAFs (Figure 2B). In the further investigation of relationships between hub genes and the immune microenvironment of OvC, we focused on IL-33. The ESTIMATE algorithm was performed to assess components in the TM of patient samples ranked by the mRNA level of IL-33. Those patients with relatively high IL-33 expression also owned higher stromal score and immune score (Figure 2C).

**FIGURE 2:** Investigating the relevance between CAF signatures and OvC immune microenvironment. **(A)** Heatmap shows the correlations between CAF signatures and hub genes of CAFs in OvC data sets. **(B)** Correlations between CAF signatures with interleukins, chemokines, and other cytokines. **(C)**TM scores in OvC samples ranked by the gene expression of IL-33.

### 3.4 Molecular characterization of the isolated CAF and EPT from OvC

To further characterize the isolated epithelial and fibroblast cells, we performed quantitative qRT-PCR to determine the expression of several epithelial and fibroblast markers. Epithelial cells showed high expression of EpCAM, CK8, and E-cadherin, with low expression of α-SMA, FAP, and FSP-1. The expression level shown was normalized with the level of GAPDH. In contrast, the four fibroblast cells isolated from ovarian cancer showed greater expression of α-SMA, FAP, and FSP-1, with low expression of EpCAM, CK8, and E-cadherin (Figure 3A). These data suggested that we were successful in isolating relatively pure epithelial cells with their fibroblast counterparts from the ovarian cancer tissues. Immunofluorescence staining confirmed the results of qRT-PCR (Figure 3B).

**FIGURE 3:** **(A)** Expression of CAFs and epithelial markers in the primary epithelial and fibroblast cells. **(B)** CAFs and epithelial markers detected by immunofluorescence staining.

### 3.5 Abundance of ST2 and IL-33 in CAFs

Analysis of the gene expressions revealed the presence of both *ST2* and *IL-33* genes in CAFs (Figures 4A, B). qRT-PCR analysis approved not only the enhancement in *ST2* and *IL-33* mRNA expression in CAFs but also their increases in the epithelial cells (EPT) as compared to the healthy group (Figures 4C, D). Invariably, the protein expressions of ST2 and IL-33 were also significantly enhanced in TM in both CAFs and epithelial cell groups when compared with healthy groups, respectively (Figures 4E,G). However, the sST2 protein was not detected in CAFs using western blotting analysis. Concentrations of IL-33 in CAFs and EPT ranged from 13.12 to 68.67 ng/mL in OvC and from 5.24 to 32.40 ng/mL in healthy controls. Concentrations of IL-33 were significantly higher in CAFs and EPT groups than in healthy subjects (*p* < 0.05). Concentrations of sST2 in CAFs and EPT ranged from 3.12 to 11.67 ng/mL in OvC and from 0.24 to 1.40 ng/mL in the healthy group. Concentrations of sST2 were significantly higher in CAFs and EPT groups than in the healthy group (*p* < 0.05). No significant difference was observed in serum concentrations of IL-33 and sST2 between patients with OvC and healthy controls (*p* = 0.08). These findings propose that ST2 and IL-33 are attending in ovarian cancer TM, and there may be IL-33/ST2 axis activation in ovarian cancer TM in CAFs and epithelial cells (Figures 4F, H).

**FIGURE 4:** Expression of IL-33 and ST2 in CAFs. **(A,B)** Expression of *IL-33* and *ST2* genes/mRNAs in the CAFs in the patient and healthy groups as assessed by qRT-PCR. **(C,D)** Expression of *IL-33* and *ST2* genes in the epithelial cells of the patient and healthy groups as assessed by qRT-PCR. **(E)** Expression of IL-33, ST2, and sST2 protein in the CAFs of the patient and healthy groups as assessed by western blotting. **(F)** The concentration of IL-33 and sST2 was measured by ELISA assays in the CAFs, healthy, and serum. **(G)** Expression of IL-33, ST2, and sST2 protein in the epithelial cells of the patient and healthy groups as assessed by western blotting. **(H)** The concentration of IL-33 and sST2 was measured by ELISA assays in the EPT, healthy, and serum.*p < 0.05 and **p < 0.01.

### 3.6 Genetic alteration and acetylation analysis

The distribution of the IL-33 genetic alteration is presented in Supplementary Figure S1. We found that a missense mutation existed in OvC in The Cancer Atlas data, which was located at the 533^rd^ nucleotide and 171^st^ amino acid. We explored the acetylation rate of *IL-33* and *ST2* genes to learn more about the role of the IL-33/ST2 axis in CAFs, EPT, and healthy groups. Our findings demonstrated that the acetylation level of H3 histone at the IL-33 promoter was increased in CAFs, while the acetylation level of H3 histone was decreased in the EPT and healthy group. However, the acetylation level of the H4 histone of IL-33 and the acetylation level of the H3/H4 histone of ST2 were not significantly altered in all groups (Figure 5A).

**FIGURE 5:** **(A)** Acetylation rate at the promoter of IL-33 and ST2 genes in CAFs, EPT, and healthy cells. **(B)** Immunohistochemical staining of IL-33 and ST2 in the OvC tissue showed the presence of ST2 and IL-33 in both epithelial cells and cancer-associated fibroblasts. **(C)** Representative image of immunohistochemistry of α-SMA and E-cadherin (in brown) from healthy and tumor samples from OvC patients (objective ×20). Blue arrowheads indicate positive cells in healthy, black arrows heads indicate E-cadherin positive tumor cells, and red arrowheads indicate α-SMA positive stromal cells. **(D)** Contribution of the IL-33 and T2 protein. **(E)** Comparison of IL-33 and ST2 genes abundance in tumor epithelial cells and CAFs as determined by qRT-PCR. **(F)** Comparison of ST2 and IL-33 protein abundance in CAFs and epithelial cells as determined by western blotting. **(G)** Comparison of ST2 and IL-33 protein concentrations in CAFs and epithelial cells as determined by ELISA. Contribution of the IL-33 and T2 protein. Data are mean ± SEM. *p < 0.02 and **p < 0.01.

### 3.7 Distribution of IL-33 and ST2 in OvC

The content of IL-33 in the healthy ovary was limited to endothelial nuclear staining and some cytoplasmic staining in mononuclear cells and was scarcely observed in the epithelium (Figure 5B). While the content of α-SMA in the healthy ovary was limited to sub-epithelial myofibroblasts and vessels (Figure 5C), the co-expression of both markers was only observed in blood vessels (Figure 5D). In the tumor, IL-33 distribution is heterogeneous among patients, observing both nuclear and cytoplasmic staining in tumor epithelial cells, with stromal staining in fibroblast-like cells, mononuclear cells, and endothelium (Figure 5B). Co-expression of IL-33 and α-SMA in tumors with advanced invasion (higher than pT3) showed a high proportion of IL-33/α-SMA cells, suggesting that CAFs can express IL-33 in more invasive stages (Figure 5D). The ST2 content in the healthy ovary was observed mainly in mononuclear cells, being almost absent in epithelium (Figure 5B). E-cadherin distribution was only limited to the healthy epithelium and homogeneous in all samples (Figure 5C), while the co-expression of both markers in the healthy colon was not observed (Figure 5D). In tumors, ST2 expression was heterogeneous among patients, and cytoplasmic staining of epithelial tumor cells as well as in fibroblasts and mononuclear cells was in stroma (Figure 5B). Measurements by western blotting and qRT-PCR exhibited that the IL-33 and ST2 protein and gene abundance was higher in CAFs than in epithelial cells (Figures 5E, F), suggesting that CAFs are the primary site of ST2 and IL-33 expression in OvC. By using the ELISA technique, IL-33 and ST2 were found in the both CAFs and EPT. Concentrations of IL-33 and ST2 were significantly higher in the CAFs group than in the EPT group (Figure 5G).

### 3.8 Induction of IL-33 expression by inflammatory mediators in CAFs

Next, we examined the upstream signals that may regulate the IL-33 expression in CAFs at OvC. We found that inflammatory mediators pertinent to OvC or TM including LPS (1, 10, and 50 ng/mL; 24 h), SAA1 (1, 10, and 50 ng/mL; 24 h), and IL-1β (0.1, 1, and 10 ng/mL; 24 h) (50–52), all increased the IL-33 protein and gene expression in a concentration-dependent form in CAFs (Figures 6A–C). Of interest, IL-33 (50, 100, and 200 ng/mL) also induced its protein and gene expressions in CAFs in a concentration-dependent form (Figure 6D). Mechanistic studies demonstrated that the induction of IL-33 abundance by these inflammatory mediators including IL-33 itself could be completely blocked by JSH-23 (JSH; 10 μM), a blocker of NF-κB (P65) nuclear translocation (Figures 6E–H). These data suggest that the common inflammatory transcription factor NF-κB is crucial for the IL-33 expression. The IL-33 self-induction property indicates that there may be a feed-forward induction of IL-33 expression in CAFs at OvC.

**FIGURE 6:** Induction of IL-33 by LPS, SAA1, IL-1β, and IL-33 in CAFs. **(A–C)** Concentration-dependent effects of LPS (0, 1, 10, and 50 ng/mL; 24 h **(A)**) IL-1β (0, 0.1, 1 and 10 ng/mL; 24 h **(B)**), and SAA1 (0, 1, 10 and 50 ng/mL; 24 h **(C)**) on IL-33 protein and gene expression in CAFs. **(D)** Concentration-dependent effect of IL-33 (0, 50, 100 and 200 ng/mL; 8 h) on *IL-33* protein and gene expression in CAFs. **(E–H)** Blockade of LPS-, IL-1β-, SAA-, and IL-33-induced increases in IL-33 protein abundance by NF-κB inhibitor JSH-23 (JSH; 10 μM). *p < 0.05, **p < 0.01, and ***p < 0.001.

### 3.9 Effect of IL-33 abundance on inflammatory factors in CAFs

Next, we explored whether IL-33 had any impact on the expression of inflammatory factors pertinent to OvC in CAFs, including COX-2, IL-6, and IL-1β, synthesis of the rate-limiting enzyme in prostaglandin. The time course study showed that IL-33 (100 ng/mL) induced the genes encoding COX-2, IL-6, and IL-1β in the time-dependent form with maximum impacts peaked at 8 h for PTGS2 and IL1B and at 4 h for IL-6 (Figure 7A). The concentration-dependent study revealed that IL-33 (50, 100, and 200 ng/mL) induced the genes encoding IL-6, IL-1β, and COX-2 in a dose-dependent form with maximal effects observed at 200 ng/mL (Figure 7B). In addition to the gene expression, IL-33 also increased COX-2 protein abundance (Figure 7C) and the secretion of PTGS2, IL-1β, and IL-6 in CAFs (Figure 7D).

**FIGURE 7:** Effect of IL-33 on the expression of COX-2, IL-1β, and IL-6 in cancer-associated fibroblasts. **(A)** Time-dependent (0, 2, 4, 8, 12, and 24 h) induction of PTGS2, IL1B, and IL6 mRNA expression by IL-33 (100 ng/mL). **(B)** Concentration-dependent induction of PTGS2, IL1B, and IL6 gene abundance by IL-33 (0, 50, 100, and 200 ng/mL; 8 h). **(C)** Concentration-dependent induction of COX-2 protein by IL-33 (0, 50, 100, and 200 ng/mL; 8 h). **(D)** Induction of PTGS2, IL-6, and IL-1β secretion by IL-33 (100 ng/mL; 8 h). *p < 0.05, **p < 0.01, and ***p < 0.001.

### 3.10 NF-κB and MAPKs roles in the induction of COX-2, IL-1β, IL-6, and expression by IL-33 in CAFs

IL-33 (100 ng/mL; 0, 0.5, 1, 2, 4, and 6 h) treatment enhanced the JNK, p38, and ERK1/2 phosphorylation, the three members of MAPK family, in the time-dependent form with maximum impacts peaked at 2 h for JNK and at 1 h for p38 and ERK1/2 in CAFs (Figure 8A). In addition, IL-33 (100 ng/mL; 8 h) also expanded the p65 phosphorylation (Figure 8B), an NF-κB complex subunit, which could be blocked by SP600125 (SP; 20 μM), SB203580 (SB; 10 μM), and PD98059 (PD; 20 μM), the respective inhibitors for JNK, p38, and ERK1/2.

**FIGURE 8:** Phosphorylation of JNK, p38, ERK1/2, and p65 by IL-33 in CAFs. **(A)** Time-dependent effects of IL-33 (100 ng/mL) on JNK, ERK1/2, and p38 phosphorylation. **(B)** Effects of JNK inhibitor SP600125 (SP; 20 μM), ERK1/2 inhibitor PD98059 (PD; 20 μM), and p38 inhibitor SB203580 (SB; 10 μM) on IL-33 (100 ng/mL; 8 h)-induced NF-κB p65 phosphorylation. **(C)** Blockade of IL-33 (100 ng/mL; 8 h)-induced IL-1β, COX-2, PTGS2, and IL-6 production by p38 inhibitor SB203580 (SB; 10 μM). *p < 0.05, **p < 0.01, and ***p < 0.001.

Moreover, JNK, p38, ERK1/2, and NF-κB inhibition with SB (10 μM) also blocked the induction of COX-2 abundance and IL-6, PTGS2, and IL-1β secretion in CAFs by IL-33 (Figure 8C). These results indicate that IL-33 can sequentially lead to the activation of MAPKs and NF-κB pathways in CAFs to induce inflammatory factors pertinent to OvC.

### 3.11 Role of ST2 receptor in the effect of IL-33 in CAFs

To investigate the ST2 receptor’s role in the effect of IL-33 in CAFs, siRNA-mediated knockdown of ST2 was executed (Figure 9A). We found that siRNA-mediated knockdown of ST2 blocked not only the induction of COX-2, IL-1β, and IL-6 but also the induction of p65, p38, ERK1/2, and JNK phosphorylation by IL-33 (100 ng/mL) in CAFs (Figure 9B). These findings propose that these IL-33 impacts are mediated by the ST2 gene in CAFs.

**FIGURE 9:** Role of ST2 in the induction of COX-2, IL-6, and IL-1β by IL-33 in CAFs. **(A)** Effects of ST2 siRNA-mediated knockdown on the protein abundance by IL-33. **(B)** Effects of siRNA-mediated knockdown of ST2 on the induction of COX-2, IL-6, and IL-1β and phosphorylation of p38, ERK1/2, JNK, and p65 by IL-33 (100 ng/mL; 1.5 h). *p < 0.05, **p < 0.01, and ***p < 0.001.

### 3.12 IL-33 stimulates proliferation, migration, and invasion

Anti-IL-33 was used to treat Caov3, SK-OV-3 cells, and co-culture (SK-OV-3+CAFs), and it decreased the effects of cell proliferation, invasion, and migration (Figures 10A–C). These results suggested an oncogenic role for IL-33. Combining these results, it is possible to exploit IL-33 expression inhibition as a therapeutic target. To determine the impacts of CAFs on cell migration and invasion, co-cultured CAFs with SK-OV-3 were examined by CCK8 assay. As shown in Figure 10B, it was demonstrated that SK-OV-3 cells treated with CAFs containing medium have high levels of cell migration. In addition, a significant increase was also observed in invading SK-OV-3 + CAFs compared with Caov3 and SK-OV-3 cells (Figure 10C). The results revealed the promoting role of CAFs in OvC cell migration and invasion.

**FIGURE 10:** Effect of IL-33 and CAFs on cell viability, invasion, and migration. **(A)** Anti-IL-33 antibody impact on the cell viability. **(B)** Anti-IL-33 antibody impact on the cell migration of Caov-3, SK-OV-3 lines, and co-cultured SK-OV-3+CAFs. **(C)** Anti-IL-33 antibody impact on the cell invasion of Caov-3, SK-OV-3 lines, and co-cultured SK-OV-3+CAFs as assessed by CCK8, Transwell, and wound healing assays. *p < 0.05, **p < 0.01, and ^##^ *p* < 0.01.

## 4 Discussion

In this investigation, we have provided evidence that the IL-33/ST2 axis is present in ovarian CAFs, and its activation may affect the inflammatory reaction of the tumor microenvironment (TM) by increasing the induction of inflammatory elements pertinent to ovarian cancer (OvC) in both CAFs and epithelial cells. We revealed that IL-1β, IL-6, and PTGS2 were among the inflammatory factors which were induced by IL-33 via the MAPKs-NF-κB signaling pathway activation in ovarian CAFs. Since the IL-33 expression could be induced by LPS, SAA1, and IL-1β, the crucial molecules involved in both infectious and non-infectious inflammation (Keelan et al., 2003; Ye and Sun, 2015; Li T et al., 2017), we believe that our findings may carry significance in both healthy and patient groups. Notably, we found that IL-33 also induced its production in fibroblasts, indicating that there may be a feed-forward of IL-33 expression in CAFs in OvC. The important IL-33 role in OvC was endorsed by our findings that IL-33 administration could indeed induce tumor progression in the cell lines. As a substantial source of interleukins and cytokines, CAFs certainly orchestrate the composition and content of soluble substances in TM and thus contribute to tumor progression. The correlations between CAF signatures and components of the immune microenvironment implied that elevated expression of interleukins and cytokines, the enrichment of immunosuppressive macrophages, mesenchymal activation, and enhanced immunotherapy resistance were all linked to CAFs’ enriched microenvironment. There have been specific studies about IL-33 in CAFs in tumor progression. Fibroblast-derived IL-33 facilitated tumor cell intravasation and T cell-mediated tumor control (Ahirwar et al., 2018; Mariathasan et al., 2018). Also, CAFs expressed IL-33 for their tumor-supporting properties (Augsten et al., 2009; Augsten et al., 2014).

Certain ovarian functions, including ovulation and estrus cycles, cause variations in IL-33 expression (Carlock et al., 2014). According to studies, the immunological molecule that is most noticeably increased during ovulation is IL-33 (Wu et al., 2015; Larsen et al., 2018; Liu et al., 2019). Except for ovaries taken throughout the estrous cycle and during ovulation, numerous randomly selected ovaries displayed a more increased amount of IL-33 compared to other tissues (Larsen et al., 2018). This implies that IL-33 expression may also be influenced by other unidentified causes. It has been found that metastatic tumor lesions and OvC tissues express IL-33 much more than benign lesions do (Saied and El Etreby, 2017). Moreover, ST2 expression was upregulated in 87% of metastatic OvC and 66% of primary sites when compared to normal human ovarian tissue samples, which was more pronounced than the increase of the IL-33 level in 77% of metastatic ovarian tumors and 60% of primary sites (Tong et al., 2016). Another investigation has indicated that epithelial ovarian cancer patients’ poor overall survival is strongly correlated with high IL-33 and ST2 expression (Tong et al., 2016). However, as some current in-depth studies have explained, some findings suggest that IL-33/ST2 has an anticancer function that may be dependent on the TM and at particular phases of tumor progression and development (Fournié and Poupot, 2018; Shen et al., 2018; Helbig et al., 2020). Hence, it is unclear whether the IL-33/ST2 axis plays a pro- or anti-tumor role.

In this study, we demonstrated that secreted IL-33 played a crucial role in the progression of OvC by invasion, immune suppression, and inducing angiogenesis, which may clarify why there are contradictory modifications in the nuclear and secreted IL-33 abundance at OvC though we are unclear about the concurrent changes of nuclear IL-33 abundance in CAFs at the current stage. We speculate that there may be a switch of nuclear IL-33 to IL-33 secretion at OvC so that IL-33 can serve as a cytokine to exert its initiating effects through the ST2 receptor in the TM. We also found that the increase in the H3 histone acetylation of the IL-33 promoter increases the expression of IL-33 in CAFs. Although to clarify how the H3 histone acetylation impacts the IL-33 promoter, more research is required.

Additionally, we revealed that the IL-33 effect on inflammatory factors was mediated by ST2 in ovarian CAFs. ST2 is present in two main differentially spliced variants: a membrane-bound form (ST2 or ST2L), mediating the cytokine effect of IL-33, and a soluble form (sST2), which is also known as a seduction receptor inhibiting the IL-33 impact (Griesenauer and Paczesny, 2017). We also discovered that the protein expression of ST2 is enhanced in the CAFs at OvC, while the sST2 protein was undetectable, indicating that ST2 but not sST2 is predominantly expressed in ovarian TM at OvC. The important role of ST2 in mediating the IL-33 impact was illustrated by the siRNA-mediated knockdown of ST2 expression in CAFs, which substantially canceled the IL-33 effects.

The IL-33/ST2 pathway activation has been linked to the activation of MAPKs and NF-κB pathways in different cell types including osteoblastic cells, mast cells, and dendritic cells (Rincón and Davis, 2009; Mine et al., 2014; Pinto et al., 2018; McCarthy et al., 2019). Here, in this study, we also demonstrated that MAPK and NF-κB pathways underpinned the IL-33 actions in ovarian CAFs. In mammals, MAPKs could be classified into three primary subfamilies, namely, JNK, ERK, and p38, which have been demonstrated to be associated with both infection and non-infection-induced inflammatory responses (Rodriguez-Barbero et al., 2006; Arthur and Ley, 2013; Ni et al., 2022). In this regard, we found that all three MAPKs were involved in the induction of IL-6, PGE2, and IL-1β expressions by IL-33 in ovarian CAFs, further indicating a crucial role of MAPKs in the inflammatory responses of the TM at OvC. NF-κB is a key inflammatory transcription factor (Liu et al., 2017), and the transcriptional activity of NF-κB can be activated following the activation of MAPK signaling cascades (Schulze-Osthoff et al., 1997). Therefore, we also demonstrated that NF-κB was activated following the activation of MAPKs in ovarian CAFs. Given the classical function of NF-κB in the mediation of pro-inflammatory mediators’ abundance in inflammation, we suppose that there may be other IL-33-inducible pro-inflammatory mediators in addition to COX-2, IL-6, and IL-1β in CAFs of ovarian cancer. Indeed, it should be an impressive subject to investigate in the future.

## 5 Conclusion

The literature has not made significant progress in explaining how IL-33 affects ovarian cancer. In this study, we have integrated a wide array of RNA-seq data to identify hub high-traffic mRNA in ovarian cancer tissues. We have also shown that ovarian TM in CAFs and epithelial cells exhibit the IL-33/ST2 axis activation, which is linked to inflammatory responses of the TM. We also showed that compared with cancer cells, CAFs significantly promoted the proliferation, migration, and invasion of OvC cells. Therefore, IL-33/ST2 axis activation, which increases the inflammatory molecules produced in the microenvironment relevant to OvC and its levels, is associated with enhanced cell proliferation, invasion, and migration. IL-33 and its related axis or pathway could be targeted as a new therapeutic goal to slow the progression of ovarian cancer.

## Data Availability

The original contributions presented in the study are included in the article/Supplementary Material; further inquiries can be directed to the corresponding authors.

## Abbreviations

CAF, cancer-associated fibroblast; COX-2, cyclooxygenase-2; DMEM, Dulbecco’s modified eagle medium; EPT, epithelial cell; FPKM, fragments per kilo base per million mapped reads; GEO, Gene Expression Omnibus; IL-33, interleukin-33; LPS, lipopolysaccharide; OvC, ovarian cancer; PBS, phosphate buffer saline; PGs, prostaglandins; qRT-PCR, quantitative real-time polymerase chain reaction; RIPA, radioimmunoprecipitation assay; and siRNA, small interfering RNA.
